The article "Changes of Short-Term Heart Rate Variability and Vertebral Artery Magnetic Resonance Angiography in Patients with Cervical Vertigo" was retracted in 2023. Reasons: signs of a paper mill; compromised peer review; unreliable results or conclusions.

# Changes of Short-Term Heart Rate Variability and Vertebral Artery Magnetic Resonance Angiography in Patients with Cervical Vertigo

**DOI:** 10.1155/2022/9551263

**Published:** 2022-09-22

**Authors:** Yu Yin, Jianli Bu, Jian Cui, Yuhang Qian, Yibing Wang

**Affiliations:** Department of Orthopedics, Bethune International Peace Hospital, Shijiazhuang 050000, Hebei, China

## Abstract

Cervical vertigo refers to a clinical syndrome with sudden vertigo as the main symptom caused by the hemodynamic disturbance of the extracranial segment of the vertebral artery (VA) affected by cervical vertebral lesions. Small differences in pulse intervals in a patient's continuous sinus rhythm are called heart rate variability (HRV). Heart rate variability refers to the small rise and fall of instantaneous heart rate between consecutive beats and is one of the most important physiological indicators of cardiac function. Small changes between successive beats reflect some information about the heart. So, it can be used to diagnose heart disease; its parameters can be used to identify emotions. Therefore, it is possible to use the characteristics of heart rate variability to find some patterns in the high-stress state and use the computer and ECG signals to describe the high-stress state. Since the ECG signal is a universal and objective model, it is practical and convenient to use it to describe stress states. Magnetic resonance angiography (MR angiography, MRA) is a noninvasive vascular imaging method that does not require intubation and contrast agents. At present, it has been widely used in clinical practice. In order to explore the changes of short-term heart rate variability and vertebral arterial magnetic resonance angiography (MRA) in patients with cervical vertigo and their clinical significance, this paper introduces two basic analysis methods of heart rate variability and commonly used MRA techniques, TOF technology. In the analysis of heart rate variability in patients with cervical vertigo, the statistical values of time and spectrum domain parameters were found to be lower in the experimental group than in the control group1. MRA showed that the abnormal rate of VA in the PCI group and the cervical vertigo group was similar. In the RMSSD index, the male experimental group reached 29, and the control group 1 reached 22.

## 1. Introduction

Heart rate variability (heart rate variability, HRV) refers to the small difference between successive heartbeats, reflecting the fine regulation of neurohumoral factors on the cardiovascular system. Heart rate variability analysis is an economical, effective, and noninvasive detection method widely used in clinic to evaluate the regulation of cardiac sympathetic and parasympathetic nerves. It is of great value in understanding heart disease and judging the prognosis of patients. With the development and continuous progress of magnetic resonance imaging (MRI), its clinical application has become more and more extensive, and people have generated great interest in magnetic resonance angiography. Medical imaging is an important auxiliary tool for clinical diagnosis and disease treatment, which helps doctors to observe the lesions in the human body more directly and clearly. It provides great convenience for doctors to accurately diagnose the patient's condition and provide timely treatment. It not only helps to relieve patient pain, but also reduces medical costs. Magnetic resonance angiography (MRA) is considered to be a noninvasive blood vessel screening method. It can objectively display abnormal changes in the vertebrobasilar artery. It has a high degree of consistency with the DSA examination, and it has now partially replaced DSA as the best means of examining VA.

The article "Changes of Short-Term Heart Rate Variability and Vertebral Artery Magnetic Resonance Angiography in Patients with Cervical Vertigo" was retracted in 2023. Reasons: signs of a paper mill; compromised peer review; unreliable results or conclusions.

When analyzing the time and frequency domain parameters of the short-range HRV data in this study, it was found that the statistical scores of the time and frequency domain parameters were lower in the laboratory group than in the control group1. In the RMSSD index, it reached 29 in the male laboratory group and 22 in the control group 1 and 35 in the female laboratory group and 22 in the control group 1. Moreover, in control group 1, women's indicators were higher than men's. The VA status of 60 patients with cervical vertigo and 44 patients with posterior circulation ischemia (PCI) was compared by MRA examination. MRA showed that the abnormal rate of VA in the PCI group and the cervical vertigo group was similar. Both groups had abnormal manifestations such as tortuosity, dysplasia, and vascular stenosis of VA. However, in the cervical vertigo group, VA tortuosity was more common, and the proportions of male and female patients were 52% and 55%.

Whiplash dizziness is a frequent condition associated with several muscle skeletal disorders. Yet, to this day, ultrasound characteristics of the neck muscles in individuals with whiplash have not been researched. Talebi et al. investigated the size of the neck muscles in subjects with whiplash and in healthy controls. The thickness of the neck flexors and extensors was assessed by ultrasonography. Depending on the results of the study, the size of the long neck muscles may be related to the etiology of cervical vertigo. But it is not very practical [1]. Bécares et al. discussed the role of cervical spine radiography in studies of patients with vertigo. He studied cervical radiographs, CT and MRI, and radiological findings in the samples. He analyzed the demographic characteristics, psychopathology, and emergency response of vertigo of patients undergoing cervical studies. It was found that 57% of patients received cervical X-ray examination. Studies have shown that the need for cervical spine X-rays in patients with glare and dizziness is influenced by sociodemographic factors. Considering the doubt of cervical dizziness, he did not believe that the findings of X-rays contribute to the diagnosis and that cervical glare and dizziness sufferers overuse X-rays [2]. Vertigo is a common symptom in patients with cervical spondylosis, but there are not many in-depth studies on it.

The article "Changes of Short-Term Heart Rate Variability and Vertebral Artery Magnetic Resonance Angiography in Patients with Cervical Vertigo" was retracted in 2023. Reasons: signs of a paper mill; compromised peer review; unreliable results or conclusions.

Banana leaf bath (BLB) [a form of solar therapy (sunbathing)] is practiced in many naturopathic hospitals in India for the treatment of various diseases; however, little is known about its precise physiology. Therefore, Fj et al. evaluated the impact of BLB on heart rate variability (HRV) in fit subjects. The results of the study showed a significant increase in the interval among adjoining QRS wave groups or transient heart rates (RR intervals), the standard deviation of RR intervals (SDNN), and the squared and mean squaring errors (RMSSD) of the difference between neighboring normal intervals and normal intervals. The findings suggest that 30 minutes of BLB may be effective in reducing HR and improving vagal innervation of HRV in healthy individuals [3]. Elhakeem et al. compared HRV in patients with typical chest pain. After evaluation of medical history and clinical investigations, he performed ECG recordings using a Bluetooth electrocardiogram (ECG) transmitter and recipient and assessed HRV in the temporal and frequency domains. The results found that, in subjects with normal angiograms according to ECA compared to patients with coronary artery disease, Ln (pNN10), Ln (pNN20), LnLF, and LnHF had significantly higher mean ± SD. However, these statistics significant differences disappeared when adjusted for age, sex, BMI, and HR in the study groups for comparison. Thus, HRV was relatively comparable in patients with typical chest pain irrespectively of ECA results [4]. Extracting HRV features is an important research direction in the study of patients with cervical vertigo, but the results of previous studies are not convincing.

The vertebral artery (VA) usually enters the sixth transverse foramen (TF). VA sometimes goes into the fifth TF, rarely the fourth or seventh TF. Uchino et al. reported two cases of magnetic resonance (MR) angiography showing the right VA into the third TF. Coronal reformatted MR angiography source images help determine the level of VA entry into the TF. There is a risk in anterior neck surgery because the abnormal VA is located anteriorly. Therefore, correct diagnosis is important when interpreting magnetic resonance angiography of the neck. Aerobic exercise is effective in preventing cerebrovascular disease [5]. Lee et al. studied cerebrovascular changes by comparing MRA (magnetic resonance angiography) images before and after aerobic exercise. Therefore, the obtained MRA images showed that the signal intensity of ECA (external carotid artery) and STA (superficial temporal artery) increased compared with before and after aerobic exercise. However, the ICA and BA of the internal carotid artery, vertebral artery, and vertebral artery all decreased. Comparison of vessel thickness before and after aerobic exercise resulted in increased ECA and STA, while ICA, VA, and BA decreased. Changes in cerebral blood vessels during aerobic exercise were analyzed with MRA images. These data show changes in blood flow and vessel thickness after aerobic exercise. Studies have shown that aerobic exercise increases cerebral blood flow and blood vessel thickness. Therefore, aerobic exercise is expected to help prevent cerebrovascular disease [6]. The above studies conducted a detailed analysis of short-term heart rate variability and vertebral artery magnetic resonance angiography changes. It is undeniable that these studies have greatly promoted the development of the corresponding fields. We can learn a lot from methodology and data analysis. However, the research on it in the medical field is relatively few and not thorough enough, and it is necessary to fully apply these techniques to the research in this field.

The article "Changes of Short-Term Heart Rate Variability and Vertebral Artery Magnetic Resonance Angiography in Patients with Cervical Vertigo" was retracted in 2023. Reasons: signs of a paper mill; compromised peer review; unreliable results or conclusions.

## 2. Methods of Short-Term Heart Rate Variability and Vertebral Artery Magnetic Resonance Angiography in Patients with Cervical Vertigo

Cervical vertigo is a clinical syndrome in which the extracranial segment of the vertebral basilar artery is damaged due to cervical spondylosis, resulting in abnormal hemodynamics and sudden onset of vertigo as the main symptom. Along with the fast developing of computers usage and electrical housing technology, great advancement has been made in medical imaging technology in recent years [7]. Ultrasound, computerized tomography (CT), and magnetic resonance imaging (MRI) are the three main methods of medical imaging [8]. Magnetic resonance imaging has become one of the most significant methods of clinical examination and an important tool for physicians to accurately diagnose certain diseases. Compared with the other two imaging techniques, MRI has the advantages of noninvasive, all-around, multicontrast, multiparametric, and high-resolution imaging, high sensitivity to soft tissues, and flexible examination methods [9]. Magnetic resonance angiography (MRA) is a noninvasive vascular study that objectively visualizes abnormal lesions in the vertebrobasilar artery. The application of MRA in the vertebral artery has high sensitivity, specificity, and high resolution, and the image is clear. It is a new noninvasive vascular technology that provides clear and intuitive images of the entire vertebral artery bilaterally. It is most commonly used in the examination of carotid bifurcation lesions. Because the blood flow of the neck vessels is large, there is no interference from movement artifacts such as breathing, the image quality is good, and an angiogram from the origin of the carotid artery to the siphon segment can be obtained. A vertebral angiogram is an ideal test for studying cervical spine disease because it provides doctors with a wealth of information about changes in the vertebral arteries and treatment options. It has been well accepted by modern physicians [10].

The article "Changes of Short-Term Heart Rate Variability and Vertebral Artery Magnetic Resonance Angiography in Patients with Cervical Vertigo" was retracted in 2023. Reasons: signs of a paper mill; compromised peer review; unreliable results or conclusions.

The heart is the main blood-pumping organ of the human body. In order to ensure normal vital function of body tissues and organs, it needs to be beating constantly to improve blood flow and energy transfer, so it needs regular supply of nutrients and energy. Heart rate variability (HRV) refers to the instantaneous increase or decrease in heart rate between two consecutive beats. It reflects the state in which the cardiovascular system is affected by the tension and balance between the autonomic nervous system and sympathetic and parasympathetic nerves. For example, increased activity of the sympathetic nerve releases norepinephrine. It leads to an increase in heart rate, and increased activity of the vagus nerve releases acetylcholine, resulting in a decrease in heart rate. Heart rate variability measures the variability in the duration of each heartbeat [11]. Every beat of the heart involves mechanical contraction of the atria and ventricles, followed by relaxation. This process is called the cardiac cycle, and it corresponds to the electrical activity of the atria and ventricles during systole (depolarization and repolarization) and diastole (resting). Its electrical stimulation of the heart causes potential differences in different parts of the body, which can be recorded by an electrocardiograph, producing an electrocardiogram image. As shown in Figure 1, an electrocardiogram consists of several waves, such as *P*, *Q*, *R*, *S*, *T*, and *U*. Each heartbeat begins with a process of depolarization of the left atrium, forming a *P* wave on the electrocardiogram. The heartbeat of the left atrium is considered a single beat. A cardiac cycle is the time interval between two consecutive, adjacent *P* waves, as shown in the left ECG in Figure 1. From the sensor's point of view, the change in heart rate should be mainly determined by the PP interval. However, since it is difficult for the ECG sensor to detect the P wave, the RR interval is usually used, as shown in the right ECG in Figure 1 [12].

The article "Changes of Short-Term Heart Rate Variability and Vertebral Artery Magnetic Resonance Angiography in Patients with Cervical Vertigo" was retracted in 2023. Reasons: signs of a paper mill; compromised peer review; unreliable results or conclusions.

Statistical methods, or mathematical statistics, include direct statistical or geometric analysis of the time-series signals of sinus-paced RR intervals, where the RR interval values are arranged in chronological or periodic order [13]. The results of time-series analysis are generally used to describe the magnitude of HRV over longer periods of time (e.g., 24 hours) and to provide information on the role of the autonomic nervous system in regulating heart rate. The clinical value of HRV was assessed by calculating a series of mathematical and statistical indices of the RR interval. There are many indices and methods, of which the most widely used is descriptive [14].

(1) SDNN of the normal sinus RR interval, that is, the standard deviation of the overall mean of all normal sinus RR intervals (or NN intervals) within 24 hours, is calculated as follows.
  (1) $$\begin{array}{c} SDNN=\sqrt{\frac{1}{N}\overset{N}{\underset{i=1}{\sum }}{\left(RR_{i}-\bar{RR}\right)}^{2}.} \end{array}$$
Among them, *N* is the total number of normal pulses, RR_*i*_ is the 1st RR cycle, and $\bar{RR}$ is the average of the RR intervals of the *N* pulses. The larger the normal deviation, the larger the heart rate variability and vice versa. The normal value is > 100 ms, and if < 50 is considered abnormal, it indicates a significant decrease in heart rate variability.
(2) The standard deviation of the mean of all consecutive 5-minute serial sinusoidal periods, SDANN, is used to estimate the HRV component over a long period (24 hours). It includes estimates of the slowly changing long-term components of HRV. It divides 24 hours into 288 5-minute periods, calculates the mean RR interval for each 5-minute period, and calculates the standard deviation of these 288 mean RR intervals [15].
Calculation is as follows:
  (2) $$\begin{array}{c} S_{288}=\sqrt{\frac{1}{288}\overset{288}{\underset{i=1}{\sum }}{\left(\bar{RR_{i}}-{\bar{RR}}_{5\;\min}\right)}^{2}.} \end{array}$$
$\bar{RR_{i}}$ is the mean of the *i*-th 5 min R-R interval and ${\bar{RR}}_{5min}$* is the mean of the 288-th *$\bar{RR_{i}}$. The normal value is usually greater than 100 ms, and if it is less than 50 ms, it is abnormal.
(3) The mean square root RMSSD of the continuous values of the adjacent normal cardiac cycles of the adjacent atrium is calculated as follows.
  (3) $$\begin{array}{c} RMSSD=\sqrt{\frac{1}{N-1}\overset{N-1}{\underset{i=1}{\sum }}{\left(RR_{i+1}-RR_{i}\right)}^{2}.} \end{array}$$
*N* is the total number of normal heartbeats, and RR_*i*_ and RR_*i*+1_ are the lengths of two adjacent sinus cycles. RMS values were used to estimate the parameters of the short-range HRV and had a normal value 27 ± 12.

A magnetic resident angle imaging is a technique for vascular imaging based on magnetic resonance imaging. Due to the flexibility of MRI, MR angiography is subdivided into the contrast-enhanced MR angiography and noncontrast-enhanced MR angiography. This is the difference between needing and not needing to inject a contrast agent [16]. In noncontrast MRI, different imaging sequences can be used to obtain contrasting images of clear and dark blood, providing valuable diagnostic information from different perspectives. In MR angiography, blood flow interferes with MR signals [17]. To avoid this effect, a new gradient waveform, commonly referred to as a velocity compensation technique, had to be developed.

The article "Changes of Short-Term Heart Rate Variability and Vertebral Artery Magnetic Resonance Angiography in Patients with Cervical Vertigo" was retracted in 2023. Reasons: signs of a paper mill; compromised peer review; unreliable results or conclusions.

TOF is currently the most widely used noncontrast-enhanced MRA technique due to its excellent resolution of stenosis, obstruction, etc. It is widely used in clinical studies of intracranial vascular disease [18]. The imaging principle of TOF is to use the special “flow effect” of MR. TOF is based on the effect of the gradient waveform on the MR signal. TOF relies on the effect of blood flow, so circulating blood and immobile tissue are not exposed to the same number of radio frequency (RF) pulses. The result is a stark blood contrast [19].

TOF is a noncontrast-enhanced MRA technique based on SPGR (Spoiled Gradient Echo) sequence. To obtain MR images, several RF excitations are usually required, and the magnetization vector is excited once per repetition time (RT). The longitudinal magnetization vector never fully recovers until the relaxation time T1 << TR of the tissue longitudinal magnetization vector is reached, resulting in a loss of signal, a phenomenon known as partial or simple saturation [20]. However, at the technical level of TOF, the spatial resolution of the direction is low, the voxels are large.

In the SPGR sequence used in the TOF technique, the relationship between the magnetic resonance signal S, T1, TR, and reversal angle (FA) is expressed by the following formula:

(4) $$\begin{array}{c} X=\frac{R_{0}\sin\;\alpha \text{(}1-e^{-TR/T1}}{1-\cos\;\alpha e^{-TR/T1}}e^{-TE/{T2}^{*}}=R_{0}\sin\;\alpha f_{1}e^{-TE/{T2}^{*}}, \end{array}$$

where *f*_1_ is the unitless ratio representing the longitudinal magnetization vector at equilibrium and *R*_0_ is the original longitudinal magnetization vector at equilibrium. From formula (4), it can be concluded that if the magnetization vector is excited by *j*(*j*) radio frequency, the steady-state magnetization vector expression is

(5) $$\begin{array}{c} X_{j}=R_{0}\sin\;\alpha \left[f_{1}+{\left(\cos\;\alpha e^{-TR/T1}\right)}^{j-1}\left(1-f_{1}\right)\right]e^{-TE/{T2}^{*}}\text{.} \end{array}$$

Thus,

(6) $$\begin{array}{c} \left(1-\cos\;\alpha e^{-TR/T1}\right)<1\text{.} \end{array}$$

Static tissue can be assumed to receive an infinite number of stimulation pulses, while blood flow can be assumed to receive *j* stimulation pulses, and *j* is relatively small because it flows out of the imaged FOV over a certain time. Based on the above assumptions, the flow-dependent signal enhancement (FRE) can be derived by the following formula.

(7) $$\begin{array}{c} X_{FRE}=X_{j}-X_{\infty }=R_{0}\sin\;\alpha \left[f_{1}+{\left(\cos\;\alpha e^{-TR/T1}\right)}^{j-1}\left(1-f_{1}\right)\right]e^{-TE/{T2}^{*}}\text{.} \end{array}$$

Formula (7) shows that *X*_*FRE*_ decreases monotonically with increasing *j*, so when TR and slice thickness are constant, faster blood flow will decrease *j*, thereby increasing *X*_*FRE*_, the contrast between blood flow and background. Therefore, the TOF image layer is always chosen to be perpendicular to the direction of blood flow. When the blood flow is fast enough that the blood flow in the imaging FOV is not stimulated with each stimulation, the maximum *X*_*FRE*_ that can be achieved is

(8) $$\begin{array}{c} {X_{FRE}}_{\max}=X_{j}-X_{\infty }=R_{0}\sin\;\alpha \left(1-f_{1}\right)e^{-TE/{T2}^{*}}. \end{array}$$

When *j* is constant, the value of TR/T1 decreases and *X*_*FRE*_ increases, because when TR/T1 decreases, so does the static organized sign *X*_*∞*_.

The article "Changes of Short-Term Heart Rate Variability and Vertebral Artery Magnetic Resonance Angiography in Patients with Cervical Vertigo" was retracted in 2023. Reasons: signs of a paper mill; compromised peer review; unreliable results or conclusions.

The relationship between *X*_*FRE*_ and the reversal angle *θ* can be derived from formula (7), as shown in Figure 2:

(9) $$\begin{array}{c} m\left(t\right)=m_{0}+v_{m}t, \end{array}$$

where *m*_0_ is the initial position at *t* = 0 and *v*_*m*_ is the uniform velocity, and these spins will be subjected to the changing magnetic field.

As shown in Figure 3, the total phase accumulation during the read gradient is

(10) $$\begin{array}{c} \varphi \left(t\right)=\left(-\int_{0}^{\tau }\omega \left(t\right)dt\right)+\left(-\int_{\tau }^{3\tau }\omega \left(t\right)dt\right)=-\beta Hm_{0}\left(t-2\tau \right)-\frac{1}{2}\beta Hv_{m}\left(t^{2}-\tau^{2}\right)\tau \leq t\leq 3\tau \text{.} \end{array}$$

Now, take the echo moment as time zero, even if

(11) $$\begin{array}{c} t^{\prime }=t-2\tau \text{.} \end{array}$$

Then,

(12) $$\begin{array}{c} \varphi \left(t^{\prime }\right)=-\beta H\left(m_{0}+2v_{m}\tau \right)t^{\prime }-\beta Hv_{m}\tau^{2}-\frac{1}{2}\beta Hv_{m}t^{\prime 2}\tau \leq t^{\prime }\leq \tau \text{.} \end{array}$$

Rewrite the formula with the static term *s* and the velocity term *v*; that is,

(13) $$\begin{array}{c} \varphi \left(t^{\prime }\right)=\varphi_{s}\left(t^{\prime }\right)+\varphi_{v}\left(t^{\prime }\right)\text{.} \end{array}$$

We can get

(14) $$\begin{array}{c} \varphi_{s}\left(t^{\prime }\right)=-\beta Hm_{0}t^{\prime }\text{,}\\ \varphi_{v}\left(t^{\prime }\right)=-\frac{1}{2}\beta Hv_{m}\left(t^{\prime 2}+4\tau t^{\prime }+2\tau^{2}\right)\text{.} \end{array}$$

The phase characteristics of *φ*_*s*_(*t*′) and *φ*_*v*_(*t*′) are shown in Figure (b), showing that the phase of the static spin is zero at the echo. However, the moving spin does not converge at the echo time (*t*′=0), and the phase of the uniform spin at the echo time in the *t*′ coordinate system is

(15) $$\begin{array}{c} \varphi_{v0}=\varphi_{v}\left(0\right)=-\beta Hv_{m}\tau^{2}\text{.} \end{array}$$

With the computerization of medical equipment and the continuous improvement of medical information management systems in large and medium-sized hospitals, the DICOM (Digital Imaging and Communication Medicine) protocol was developed. Different models of equipment from different manufacturers, and thus different image formats, pose a major challenge to hospital PACS systems because it is difficult to fully utilize the resources of different equipment. The media storage strategy includes the compatibility matrix of medical images and related devices, as shown in Figure 4; the top-level service is the service provided by the DICOM standard in practical applications. These services are at the highest level and include a service group and an IOD information object. The IOD in the SOP contains a lot of properties. The service group provides media storage services and a set of DIMSE message service elements.

In DICOM format files, a dataset consists of a specific sequence of data elements. The data elements that it contains are its main components. As shown in Figure 5, the data element consists of four parts: name, data description VR, data length VL, and data field. Each field is defined as follows.

BMP image and DICOM image files can be converted.

After understanding the images in BMP format and DICOM format, it is easy to know that, after the DICOM image is converted into a BMP image, the BMP image only contains a part of the DICOM format image. It lacks some information features in DICOM, such as examination type information and patient information that need to be manually added in BMP format images. This missing information can be added manually during information collection or added to the images from the patient's database. Even if this cannot add all the information, some information still needs to be obtained from the influencing device, such as the window level, window width, and pixel space ratio of the current image. The image in DICOM format converted to the image in BMP format is shown in Figure 6.

The article "Changes of Short-Term Heart Rate Variability and Vertebral Artery Magnetic Resonance Angiography in Patients with Cervical Vertigo" was retracted in 2023. Reasons: signs of a paper mill; compromised peer review; unreliable results or conclusions.

## 3. Experimental Design of Short-Term Heart Rate Variability and Changes in Vertebral Artery Magnetic Resonance Angiography

In this paper, in order to study the changes of short-term heart rate variability and vertebral artery magnetic resonance angiography, the research subjects and groups are shown in Tables 1 and 2.

1. Experimental group: this article selected 62 patients with cervical vertigo who were admitted at a central hospital from January 2018 to February 2019. Among them, there were 31 males and 29 females; the disease duration ranged from 1 h to 2.5 years, with an average of 1.2 years. The clinical manifestations are paroxysmal or orthostatic dizziness, nausea, vomiting, limb weakness, ataxia, even sudden fainting, temporary deafness, and blindness. All patients underwent routine cervical spine X-ray and MRJ and MRA examinations.
2. Healthy control population: 55 normal people whose gender and age were matched with the cervical vertigo cases were recruited, and the exclusion criteria were the same as the patient group. At the same time, those with any symptoms of vertigo were excluded.
3. PCI group: patients with posterior circulation infarction and transient ischemic attack (TIA) admitted at our department during the same period were confirmed by head CT or MRI, 30 males and 25 females; the disease duration was from 1 hour to 2.5 years, with an average of 1.2 years.

For ease of analysis, 31 male and 29 female patients were selected for HRV analysis. Heart rate variability analysis was performed using the Cardiovascular Attitude Tester (CVFD-I). The procedure was performed while the subjects were at rest. The computer automatically calculates the heart rate variability index for 5 minutes: very low frequency power (VLF0-0.04 Hz), low frequency power (LF 0.04–0.15 Hz), high frequency power (HF 0.15–0.40 Hz), low/high frequency power (LF/HF), normalized low frequency power (LFn), and normalized high frequency power (HFn).

Individual measures for cyclical changes are explained as follows. Entropy describes the nonlinear complexity of a set of RR intervals. As far as information theory is concerned, the sensitivity of the initial value of chaotic motion means that the system is constantly producing information. So, the entropy metric is used to measure the speed of information dissemination or the speed of information flow. Chaos is bounded, not unlimited, and fluctuating. Blood pressure and heart rate per heartbeat are delayed in recovery due to the complex control mechanisms of the autonomic nervous system. When the heart is young and healthy, changes in heart rate are an unpredictable chaotic process. On the other hand, regularity of behavior increases with age and disease, which means that the complexity of the system decreases. An increase in action entropy implies a corresponding increase in self-regulation capacity and a decrease in the variability of responses to external stimuli under different conditions.

The article "Changes of Short-Term Heart Rate Variability and Vertebral Artery Magnetic Resonance Angiography in Patients with Cervical Vertigo" was retracted in 2023. Reasons: signs of a paper mill; compromised peer review; unreliable results or conclusions.

Time domain analysis of HRV mainly reflects the overall magnitude of HRV, and frequency domain analysis can be used to determine the role of sympathetic and vagus nerves in heart rate regulation. Since heart rate variability can form the frequency curve of the ECG, the Fourier transform can be used to generate the power spectral density curve shown in Figure 7. From this, the power in the relevant frequency range can be calculated and the value of each HRV parameter in that frequency range can be calculated.

Dizziness is a common symptom in patients with cervical spondylosis. Dizziness can occur in both basal cervical spondylosis and sympathetic cervical spondylosis, often as a result of sudden vertigo after falling pillows and rapid head rotation. The VA status of 61 patients with cervical vertigo and 54 patients with posterior circulation ischemia (PCI) was compared by MRA. In this paper, Neusoft 0.23T permanent magnet MRI scanner, neck coil, and MRA 2DT sequence were used, and the scanning range included cervical 1–7 vertebral bodies.

## 4. Data of Short-Term Heart Rate Variability and Vertebral Artery Magnetic Resonance Angiography

For the short-range data, the root mean square RMSSD of the continuous adjacent normal sinus cardiac cycle values of the time domain parameters and the frequency domain parameters of the total frequency power TP, low frequency power LF, high frequency power HF, and the ratio of low frequency power to high frequency power are shown in Figure 8.

The parameter values of the two teams were compared, and the findings revealed that the parameters of the experimental group were below those of the control group 1 in both time and frequency domains. Regarding the RMSSD index, the males in the experimental group scored 29 points and the control group 1 scored 22 points; the females in the experimental group scored 35 and the control group 1 scored 22. In control group 1, the index of the female group was higher than that of the male group. Indices such as RMSSD, pNN50%, and HF reflect the activity of the vagus nerve. The decrease indicates that the activity of the vagus nerve is reduced, the sympathetic nerve is dominant, and the threshold of ventricular fibrillation is lowered, which is easy to induce malignant arrhythmia. It is a disadvantage. Conversely, its exponential increase indicates increased parasympathetic tone. To some extent, LF/HF is a direct indicator of altered sympathetic and vagal balance, and an increase in LF/HFH indicates a predominance of the sympathetic nervous system. It is a disadvantage that increases the likelihood of malignant cardiac events.

The article "Changes of Short-Term Heart Rate Variability and Vertebral Artery Magnetic Resonance Angiography in Patients with Cervical Vertigo" was retracted in 2023. Reasons: signs of a paper mill; compromised peer review; unreliable results or conclusions.

Comparison of cervical vertigo and MRA abnormalities in PCI patients is shown in Figure 9.

MRA showed that the abnormal rate of VA in the PCI group and the cervical vertigo group was similar and the patients in both groups had abnormal manifestations such as tortuosity, dysplasia, and vascular stenosis. However, in the cervical vertigo group, VA tortuosity was more common, and the proportions of male and female patients were 52% and 55%. The incidence of vascular tortuosity was significantly higher than that in the PCI group, and the incidence of vascular stenosis was significantly lower than that in the PCI group (all *P* < 0.01). The main abnormality in PCI patients was vascular stenosis (male and female patients: 32% and 31%). It is common in the VA origin, intracranial segment, VA origin, intracranial segment, and stenosis of the basilar artery, which can cause hypoperfusion in the vertebrobasilar blood supply area. Patients with VA dysplasia on one side had low blood flow velocity in the affected VA and experienced a higher number of vertigoes after head and neck movements than the control group obviously.

Patients in the study group underwent CT-guided rotation and repositioning maneuvers. Statistical observation and comparison of cervical vertebral artery caliber and blood flow index before and after treatment in the two groups are shown in Tables 3 and 4.

From the analysis of Tables 3 and 4, it can be seen that the cervical vertebral artery caliber and average blood flow velocity have significantly changed after treatment in patients with cervical vertigo, which greatly reduces the distance from normal healthy people.

## 5. Conclusion

Heart rate variability is a noninvasive method commonly used in clinical practice to assess the autonomic function of the heart. It reflects the activity of the autonomic nervous system and the state of balance and coordination by continuously measuring the degree of change in the RR interval of the sinus node heart rate. The heart rate of normal individuals fluctuates at rest. Factors that influence heart rate fluctuations include enhanced cerebral nerve activity, automatic rhythmical activities of the central nervous system, respiratory activity, and cardiovascular reflexes triggered by pressure and chemical sensors. Reduced HRV reflects changes in autonomic nervous system regulation of the cardiovascular system, resulting in increased excitability of the sympathetic nervous system and reduced parasympathetic nervous system activity, leading to cardiovascular events. This study confirmed that heart rate variability was significantly lower in patients with cervical vertigo compared to age- and sex-matched normal controls. Magnetic resonance angiography is a technique used to visualize vascular characteristics and blood flow signals. This study found that, in the patients with VA dysplasia, the VA blood flow velocity on the affected side was low and the number of dizziness incidences after head and neck exercise was significantly higher than that of the control group. The role of magnetic resonance angiography in the diagnosis and treatment of vascular disease will become increasingly evident. With its advantages of being economical, efficient, and noninvasive, medical imaging plays an important role in the development of modern medicine and in the diagnosis and treatment of clinical diseases.

The article "Changes of Short-Term Heart Rate Variability and Vertebral Artery Magnetic Resonance Angiography in Patients with Cervical Vertigo" was retracted in 2023. Reasons: signs of a paper mill; compromised peer review; unreliable results or conclusions.

## Figures and Tables

**Figure 1:** ECG waveform location of HRV data.

**Figure 2:** Relationship between excitation angle and *X*_FRE_ in TOF technology (a) represents the case of TR/T1 = 0.01, and (b) represents the case of TR/T1 = 0.1. *j* represents the number of stimulation pulses received by circulating blood within the FOV imaging area. In MRI, the location of proton populations in resting tissue is relatively constant, but the location of proton populations in circulating blood is constantly changing, which inevitably affects MRI signals. An example of flow in the read direction is the rotation of the flow during sampling, which simply moves in the direction of the read gradient.

**Figure 3:** Dispersion due to flow in the read direction. (a) Read gradient waveform. (b) Additional phase accumulation for uniform motion self-selection along the direction of the read gradient.

**Figure 4:** DICOM information model.

**Figure 5:** DICOM dataset and data element structure.

**Figure 6:** Image conversion process.

**Figure 7:** HRV power spectral density.

**Figure 8:** Short-range HRV analysis.

**Figure 9:** Comparison of abnormal MRA between cervical vertigo and PCI patients (%).

**Table 1:** Age comparison between experimental group and control group.

Group		Number of cases	Age
Experimental group	Male	31	32.25 ± 7.54
	Female	29	31.95 ± 4.85
Control group 1 (healthy people)	Male	30	31.75 ± 6.78
	Female	25	33.85 ± 5.62
Control group 2 (PCI group)	Male	22	32.55 ± 5.88
	Female	22	33.85 ± 5.21

The article "Changes of Short-Term Heart Rate Variability and Vertebral Artery Magnetic Resonance Angiography in Patients with Cervical Vertigo" was retracted in 2023. Reasons: signs of a paper mill; compromised peer review; unreliable results or conclusions.

**Table 2:** General information of patients in the experimental group.

Classification of cervical vertigo	Male	Female
Vertebral artery type	19	14
Vertebral artery type (percentage)	61.3%	48.3%
Sympathetic type	12	15
Sympathetic type (percentage)	38.7%	51.7%

**Table 3:** Cervical vertebral artery caliber in treated patients.

	Caliber of the left cervical conus arteriosus	Caliber of the right cervical conus arteriosus
Before treatment	2.82 ± 0.12	2.05 ± 0.38
After treatment	3.59 ± 0.35	3.55 ± 0.28
Control group 1 (healthy people)	3.97 ± 0.39	4.01 ± 0.22

**Table 4:** Average blood flow velocity of patients before and after treatment.

	Mean blood flow velocity in the left cervical conus arteriosus	Mean blood flow velocity in the right cervical conus arteriosus
Before treatment	34.52 ± 11.01	32.05 ± 10.8
After treatment	45.19 ± 0.99	49.55 ± 10.28
Control group 1 (healthy people)	49.97 ± 0.97	49.01 ± 11.22

## Data Availability

No data were used to support this study.
